# The Relationship between the Mean Platelet Volume and Carotid Atherosclerosis and Prognosis in Patients with Acute Cerebral Infarction

**DOI:** 10.1155/2020/6685740

**Published:** 2020-12-30

**Authors:** Min Xu, Xiao-ying He, Pan Huang

**Affiliations:** ^1^Department of Neurology, The Second People's Hospital of Deyang City, No. 340 Minjiang West Road, Deyang, Sichuan, China; ^2^Department of Neurology, The Affiliated Hospital of Southwest Medical University, No. 25 Taiping Street, Luzhou, Sichuan, China; ^3^Department of Neurology, People's Hospital of Deyang City, No. 173 TaiShan North Road, Deyang, Sichuan, China

## Abstract

**Objective:**

To investigate the relationship between mean platelet volume (MPV) level and carotid atherosclerosis and prognosis in patients with acute cerebral infarction*. Methods*. A retrospectively included 160 patients with acute cerebral infarction classified by TOAST classification as aortic atherosclerosis as the observation group. To analyze the relationship between MPV and carotid atherosclerosis, and use receiver operating characteristic (ROC) curves to analyze the role of MPV in predicting the prognosis of acute cerebral infarction in the observation group, grouping patients with different MPV by cut-off value, and analyze the differences in factors between the two groups of patients.

**Results:**

MPV has a positive correlation with carotid atherosclerosis in patients with acute cerebral infarction. Multivariate logistic regression analysis revealed that increased MPV was an independent predictor of poor functional outcome in patients with acute cerebral infarction (Odds Ratio (OR): 6.152, 95% CI: 2.385-13.625, *P* < 0.01). ROC curve analysis showed that the area under the curve for MPV to predict poor prognosis was 0.868 (95% CI: 0.787-949, *P* < 0.01). The cutoff value, sensitivity, and specificity were 12.65, 76.2%, and 87.6%. Compared with patients with MPV < 12.65 at admission, patients with higher MPV levels (MPV ≥ 12.65) at admission have larger infarct size, more severe carotid artery stenosis, poor short-term prognosis, and higher mortality.

**Conclusion:**

MPV level is closely related to the degree of carotid atherosclerosis in patients with acute cerebral infarction, and it is also an independent predictor of poor prognosis in patients with acute cerebral infarction at 3 months.

## 1. Introduction

Acute cerebral infarction has a high risk of disability, death, and recurrence, which brings a serious burden to society and families [1]. Studies have shown that the important cause of acute cerebral infarction is carotid atherosclerosis. There are various screening methods for carotid atherosclerosis [2]. High-resolution CT angiography and digital subtraction angiography have high accuracy and specificity, but their price is more expensive; they are invasive examinations and have not yet been widely carried out. Doppler color ultrasound examination is convenient, fast, affordable, and suitable screening for large-scale carotid atherosclerosis. Platelets are the pathological basis of carotid atherosclerosis; mean platelet volume (MPV) is an important marker reflecting platelet activation and function [3, 4]. MPV is closely related to a variety of cardiovascular diseases or risk factors. It has been found that MPV may be related to the severity and prognosis of coronary artery disease [5, 6, 7]. At present, there are no obvious reports on the relationship between MPV and carotid atherosclerosis in patients with acute cerebral infarction and the prognostic value of patients. Therefore, this study aimed to explore the relationship between peripheral blood MPV and carotid atherosclerosis in patients with acute cerebral infarction and its predictive value.

## 2. Objects and Methods

### 2.1. Research Object

160 patients with acute cerebral infarction hospitalized from January 2013 to December 2019 in the Department of Neurology of our hospital were selected as the observation group, of which 80 were male. There were 80 females: age (44-89) years, average 67.27 ± 9.48 years old, 104 patients with a history of hypertension, and 21 patients with a history of diabetes.

The following are the inclusion criteria: (1) all patients were confirmed to be patients with cerebral infarction by cranial CT/MRI [8], (2) were admitted to the hospital within 1 week of onset, and (3) were all first attacks. The following are the exclusion criteria: (1) patients with severe liver failure or acute or chronic renal insufficiency; (2) patients with abnormal thyroid function, (3) patients diagnosed with malignant tumors; (4) patients with a history of myocardial infarction or severe heart disease patients with disease; (5) are taking lipid-lowering drugs and vitamin preparations; (6) other chronic wasting diseases, recent history of infection, and history of surgical trauma; (7) patients who lost follow-up; and (8) patients with missing test results. The research protocol was reviewed and approved by the ethics committee of our hospital, and informed consent was obtained from patients and their families.

### 2.2. Data Collection

The collected general and clinical data of all patients include age, gender, history of hypertension, history of diabetes, follow-up methods, and follow-up results. Hypertension is defined as having been previously diagnosed with hypertension or taking antihypertensive drugs regularly or having systolic blood pressure ≥ 140 mmHg and/or diastolic blood pressure ≥ 90 mmHg measured at least twice on different days of admission. Diabetes is defined as having previously diagnosed diabetes or taking hypoglycemic drugs regularly, or random blood glucose > 11.1 mmol/L, or rapid fasting blood glucose test > 7.0 mmol/L at the time of admission.

### 2.3. Carotid Artery Examination and Classification

All subjects underwent a Doppler ultrasound examination within 3 days of admission. Sonographers in our hospital used the HDI-5000 color Doppler ultrasound system (probe frequency 7-10 MHz) produced by an American ATL company to perform the examination. Observe both sides of the carotid artery (common carotid artery, bifurcation and internal carotid artery), vascular shape, intima-media thickness, the presence or absence of atherosclerotic plaque in the blood vessel (if there is atherosclerotic plaque, observe and record its location and size and morphology), and whether there are stenosis and the degree of stenosis (for multisegment stenosis, take the most severe part of the stenosis). The average value of the bilateral carotid arteries reflects the degree of thickening of the carotid media. The definition of carotid IMT is the distance between the lumen intima interface and the media adventitia interface.

### 2.4. MPV Determination

For all the included subjects, 3 ml of fasting venous blood was collected before using antiplatelet drugs, placed in a precooled EDTA anticoagulant tube, and submitted for examination within 2 hours. The laboratory physician of our hospital will perform the test. The experiment is fully automated. The blood cell analyzer strictly follows the operating procedures of the instructions to detect the peripheral blood MPV level of patients with acute cerebral infarction.

### 2.5. Determination of Cerebral Infarct Area

Calculate the maximum slice diameter of the infarct on the head CT or MRI: <1.5 cm is a small-area cerebral infarction (lacunar infarction), 1.5-5.0 cm is a medium-area cerebral infarction, and >5.0 cm is a large-area cerebral infarction.

### 2.6. Follow-Up and Grouping

After 3 months of onset, follow-up by telephone or outpatient service, evaluate the functional prognosis of the patients according to the mRS score and group them according to the prognosis of the patients. mRS score ≤ 2 is the good prognosis group, and mRS score > 2 is the poor prognosis group. Analysis of the impact on patient prognostic factors.

### 2.7. Evaluation Standard

Carotid artery IMT < 1.0 mm is normal; IMT ≥ 1.0 mm or plaque formation is regarded as abnormal; the degree of carotid artery stenosis is divided into [9]: (1) mild stenosis: the stenosis rate is 1%-49%, and the grayscale image shows local plaque is formed, the tube diameter is relatively reduced, and the blood flow has no obvious change; (2) moderate stenosis: the stenosis rate is 50%-69%, the blood flow velocity in the stenosis section increases, and the pathological vortex is formed in the distal section of the stenosis; (3) severe stenosis: the stenosis rate is 70%-99%, the blood flow velocity in the stenosis segment is further increased, the velocity in the proximal segment of the stenosis is relatively reduced, and the blood flow signal of vortex and turbulence appears in the distal segment; and (4) vascular occlusion: the blood flow signal disappeared without blood flow.

### 2.8. Statistical Methods

Statistical analysis was performed using the SPSS 17.0 Chinese version statistical software. The measurement data are expressed as mean ± standard deviation, independent sample *t*-test is used for comparison between two groups, single-factor analysis of variance is used for multiple group comparison, and Pearson correlation analysis is used for correlation analysis. By constructing a receiver operating characteristic (ROC) curve and calculating the area under the curve (AUC) to evaluate the predictive ability of MPV for poor prognosis, at the same time, according to the cutoff value of MPV, all patients are divided; the difference in factors between patients with different MPV level groups was analyzed by univariate analysis for groups less than the cutoff level and greater than or equal to the cutoff level. The difference was statistically significant with *P* < 0.05.

## 3. Results

### 3.1. Comparison of MPV Levels in Patients with Acute Cerebral Infarction with Different Degrees of Carotid Artery Stenosis

The MPV levels of patients with acute cerebral infarction with different degrees of carotid artery stenosis were compared as shown in Table 1, in which the MPV levels of the mild and moderate to severe stenosis groups were compared with those of the IMT normal group, and the MPV levels of the moderate and severe stenosis group were compared with those of the mild and moderate stenosis group; the differences were statistically significant (*P* < 0.05).

### 3.2. Comparison of MPV Levels of Acute Cerebral Infarction in Different Areas

The comparison of MPV levels of different carotid artery stenosis in patients with acute cerebral infarction is shown in Table 2. There were statistically significant differences in peripheral MPV among patients with different infarction areas (*P* < 0.05).

### 3.3. Correlation between Peripheral Blood MPV Level and the Degree and Areas of Carotid Artery Stenosis in Patients with Acute Cerebral Infarction

Pearson correlation analysis showed that MPV was positively correlated with the degree of carotid artery stenosis (*r* = 0.531, *P* < 0.05), and MPV was positively correlated with cerebral infarct areas (*r* = 0.786, *P* < 0.05).

### 3.4. Follow-Up Results

At the 3-month follow-up, 137 patients (85.6%) had a good prognosis and were included in the good prognosis group; 23 patients (14.4%) had a poor prognosis and were included in the poor prognosis group.

### 3.5. Univariate Analysis Results of General and Clinical Data of Patients in the Good Prognosis Group and Poor Prognosis Group

The results of the univariate analysis showed that the two groups of patients had statistically significant differences in age, admission infarct size classification, carotid artery stenosis, infarct location, red blood cell count at admission, hemoglobin, and red blood cell distribution width MPV (all *P* < 0.05) Table 3.

### 3.6. Multivariate Logistic Regression Analysis Results of Factors Affecting Poor Prognosis

The results show that infarct size and MPV are independent factors affecting the prognosis of patients with acute cerebral infarction, and increased infarct size and MPV are risk factors for poor prognosis in patients with acute cerebral infarction Table 4.

### 3.7. ROC Curve Analysis of MPV's Ability to Predict Poor Prognosis of Acute Cerebral Infarction

The results showed that the AUC of MPV for predicting the poor prognosis of acute cerebral infarction was 0.868 (95% CI: 0.787-0.949, *P* < 0.01), indicating that MPV has a better predictive ability for the prognosis of acute cerebral infarction. Calculate the cutoff value and select 12.65 as the critical value. When MPV ≥ 12.65, the sensitivity of MPV to predict poor prognosis is 76.2%, and the specificity is 87.6% Figure 1.

### 3.8. Comparison of Clinical Data of Patients in Different MPV Groups

The results showed that patients with higher MPV (MPV ≥ 12.65) at admission had larger infarct size and more severe carotid artery stenosis (all *P* < 0.05, Table 5). There were statistically significant differences in the 3-month mRS scores and mortality between the two groups (all *P* < 0.05, Figure 2).

## 4. Discussion

Cerebral infarction is a group of syndromes that is caused by the sudden decrease or cessation of blood flow in the local blood supply arteries of the brain tissue, causing ischemia and hypoxia of the brain tissue in the blood supply area of the responsible blood vessel, leading to necrosis and softening of the brain tissue, and accompanied by corresponding neurological deficits. The carotid artery is the main blood supply artery of the brain. Once atherosclerosis causes stenosis, it can lead to cerebral infarction.

Platelets have been known as the pathological basis of atherosclerosis for a long time. It runs through atherosclerosis. It can be said that it is the promoter and inducer of atherosclerosis [10, 11, 12]. MPV stands for the average platelet size; a number of cardiovascular disease trials have confirmed that the MPV of the experimental group is significantly higher than that of the normal control. For example, MPV is positively correlated with the degree of coronary artery disease [13]. It also has predictive value for the prognosis of percutaneous coronary intervention [14], suggesting that MPV may become an important predictor of the occurrence and prognosis of cardiovascular and cerebrovascular diseases. The mechanism may be that the larger the MPV, the platelets bind to platelet activators such as adrenaline and ADP faster, produce more coagulants and vasoactive factors, and can also express more adhesion molecules, so that hemostasis time is shorter and more easily lead to embolic events [15]. Therefore, it can be said that MPV is a marker of platelet activation and function. At present, there are not many domestic researchers engaged in this topic, and the authors conduct clinical trial observations based on this. This study shows that the MPV level in peripheral blood of patients with acute cerebral infarction is positively correlated with the degree of carotid atherosclerosis, indicating that high MPV is closely related to the occurrence and development of carotid atherosclerosis in patients with acute cerebral infarction. The possible reasons are as follows: (1) Platelets with larger MPV contain more thromboxane A2, express more glycoprotein receptors such as IIIa and IIb receptors, and have stronger chemotaxis, adhesion, and aggregation functions. In addition, the larger platelet volume can release more active factors, such as platelet factor-4 and P-selectin, which can aggravate vascular endothelial cell damage and inflammation, thereby promoting the progression of atherosclerosis and thrombosis [16]. (2) Patients with large MPV often have diseases such as hypertension, diabetes, and dyslipidemia. The synergistic effect of these factors causes vascular endothelial cell damage, causing increased secretion of interleukins and other cytokines, which in turn stimulates bone marrow hematopoietic cells to produce more platelets that become larger. The latter further promotes thrombosis and ischemic events [17]. Moreover, the ischemic tissue can also produce the above cytokines, which further promotes the bone marrow to produce more large-volume platelets [18]. (3) The larger the MPV, the platelets often exist in the form of nets, which can reduce the therapeutic effect of antiplatelet drugs and further increase the risk of thrombosis [19].

In addition, this study also showed that patients with acute cerebral infarction (MPV > 12.65) with a higher MPV level at admission had a poor short-term prognosis. Multivariate logistic regression analysis showed that patients with acute cerebral infarction at a high MPV level had a poor 3-month functional prognosis independent risk factors; the ROC curve also shows that the area under the curve for MPV to predict the poor prognosis of patients with acute cerebral infarction is 0.868. The above results all indicate that the MPV level at admission can predict the short-term prognosis of patients with acute cerebral infarction. A number of previous studies have confirmed the significance of MPV in coronary atherosclerotic heart disease, sepsis, malignant tumors, chronic kidney disease, and other diseases, all showing the correlation between high MPV levels and adverse results. In this study, the possible mechanisms of high MPV leading to poor prognosis of acute cerebral infarction are as follows: (1) High MPV may lead to endothelial dysfunction and increased inflammation. An increase in MPV indicates that the body is in a potentially proinflammatory state and further cascades. The amplified inflammatory response can lead to aggravated destruction of the blood-brain barrier, causing secondary brain damage [20, 21]. (2) The higher the risk of thrombosis in patients with high MPV levels, the greater the risk of thrombosis, which can cause repeated embolization of small blood vessels in the local brain tissue and aggravate nerves and functional impairment [22]. (3) High MPV levels are related to the balance of oxidative stress in the body, leading to the formation of high oxidative stress levels in the body, thereby weakening the deformability of red blood cells, increasing the adhesion of red blood cells and endothelial cells, and promoting thrombosis [23, 24]. The above specific mechanisms still need to be verified by subsequent basic experiments.

In short, MPV has a certain predictive value for acute cerebral infarction. In addition, MPV detection is convenient and low-cost and can be carried out by medical units at all levels. Therefore, it is useful for the prevention and prognosis evaluation of ischemic cerebrovascular in domestic (especially primary medical units) certain clinical application and reference value.

## Figures and Tables

**Figure 1:** ROC curve.

**Figure 2:** Comparison of the mRS score and fatality rate between the two groups of patients at 3 months.

**Table 1:** MPV levels in patients with different degrees of carotid artery stenosis.

Group	*N*	MPV levels
IMT normal group	29	10.31 ± 1.06
Mild stenosis group	89	11.22 ± 1.26
Moderate to severe stenosis group	42	12.90 ± 1.20
F	44.45	
*P*		<0.05

**Table 2:** MPV of patients with different infarct areas was compared.

Group	*N*	MPV
Small area group	78	10.57 ± 0.93
Medium area group	42	11.14 ± 1.16
Large area group	41	12.79 ± 1.37
F	53.63	
*P*	<0.05	

**Table 3:** Univariate analysis results of the general and clinical data of patients in the good prognosis group and poor prognosis group.

	Good prognosis group (137)	Poor prognosis group (23)	*P*
Age (years)	65.32 ± 8.75	78.88 ± 9.32	<0.01
Male (*n*, %)	74 (54.1%)	15 (65.2%)	>0.05
High blood pressure (*n*,%)	94 (68.6%)	10 (43.4%)	>0.05
Diabetes (*n*, %)	18 (13.1%)	3 (12.3%)	>0.05
Infarct size (*n*, %)			<0.01
Small area	112 (81.7%)	7 (30.4%)	
Medium and large area	25 (18.3%)	16 (69.6%)	
Carotid artery stenosis degree (*n*,%)			<0.01
Normal ITM and mild stenosis	95 (69.3%)	4 (17.4%)	
Moderate and severe stenosis	42 (30.7%)	19 (82.6%)	
Infarct site (*n*, %)			<0.01
Front loop	108 (78.8%)	5 (23.8%)	
Post loop	29 (21.2%)	16 (76.2%)	
Red blood cell count (×10^9^/l)	4.20 ± 0.52	3.78 ± 0.48	<0.01
Hemoglobin (g/l)	125.78 ± 34.28	116.41 ± 30.54	<0.01
MPV	11.03 ± 1.35	13.13 ± 1.34	<0.01

**Table 4:** Multivariate logistic regression analysis of factors influencing poor prognosis.

	OR (95% CI)	*P*
Age	1.042 (0.985-1.085)	0.126
Infarct size	14.849 (4.857-43.258)	<0.01
Red blood cell count	0.812 (0.142-4.1258)	0.589
Hemoglobin	0.998 (0.938-1.057)	0.899
MPV	6.152 (2.385-13.625)	<0.01
Infarct site	1.411 (0.415-4.802)	0.571

**Table 5:** Comparison of general and clinical data of patients with acute cerebral infarction in different MPV groups.

	MPV < 12.65 (125)	MPV ≥ 12.65 (35)	*P*
Age (years)	66.98 ± 8.86	68.30 ± 9.35	>0.05
Male (*n*, %)	62 (49.6%)	17 (48.6%)	>0.05
High blood pressure (*n*, %)	87 (69.6%)	17 (48.6%)	>0.05
Diabetes (*n*, %)	16 (12.8%)	5 (14.3%)	>0.05
Infarct size (*n*, %)			<0.01
Small area	113 (90.4%)	6 (17.2%)	
Medium and large area	12 (9.6%)	29 (82.8%)	
Carotid artery stenosis degree (*n*, %)			<0.01
Normal ITM and mild stenosis	111 (88.8%)	7 (20.0%)	
Moderate and severe stenosis	14 (11.2%)	28 (80.0%)	
Infarct site (*n*, %)			>0.05
Front loop	75 (60.0%)	20 (57.2%)	
Post loop	50 (40.0%)	15 (42.8%)	
Red blood cell count (×10^9^/l)	4.11 ± 0.48	4.24 ± 0.45	>0.05
Hemoglobin (g/l)	124.34 ± 32.64	124.76 ± 33.29	>0.05
mRS score			
≤2score	105 (84.0%)	7 (20.0%)	
>2score	17 (13.6%)	22 (62.8%)	
Death	3 (2.4%)	6 (17.2%)	<0.01

## Data Availability

All data, models, and code generated or used during the study appear in the submitted article.
